# SOX9 in Keratinocytes Regulates Claudin 2 Transcription during Skin Aging

**DOI:** 10.1155/2022/6884308

**Published:** 2022-07-31

**Authors:** Jingyan Wang, Xingyu Xie, Ying Deng, Hongqiu Yang, Xiaoshuang Du, Ping Liu, Yu Du

**Affiliations:** Affiliated Traditional Chinese Medicine Hospital of Southwest Medical University, Luzhou 646000, China

## Abstract

In order to prove that SOX9 in keratinocytes regulates claudin 2 transcription during skin aging, the skin of 8-week-old and 24-month-old mice is sequenced to obtain a differentially expressed gene SOX9. The gene is mainly expressed in keratinocytes, and it increases first and then decreases from newborn to aging. Six core sequences of SOX9 and claudin 2 are predicted from Jaspar. The double Luciferase Report shows that overexpression of SOX9 induces the full-length promoter of claudin 2 significantly and has no effect on the mutation and cleavage plasmid without SOX9 response. Claudin 2 is consistent with SOX9 in the skin of mice of different ages, and SOX9 is strongly positively correlated with claudin 2. Finally, overexpression of SOX9 and claudin 2 will delay PM2.5-induced keratinocyte senescence. The silencing of claudin 2 leads to the loss of SOX9 function. It is clearly evident that SOX9 can affect the transcription of claudin 2, which increases first and then decreases in the process of mice from newborn to aging. SOX9 inhibits proinflammatory mediators, increases antioxidant capacity, and restores keratin differentiation. It can effectively prevent melanin deposition and delay aging.

## 1. Introduction

The skin is the outermost and largest organ of the human body [1]. With the growth of age, the skin will gradually age, weaken, or lose function [2]. Aging of skin surface is reflected as cell aging at the cellular level [3]. In recent years, keratinocytes have been considered to play an extremely important role in skin aging. Keratinocytes are the main component of the epidermis and epithelial cells that can synthesize keratin. Keratin is extremely important for skin water retention, moisture retention, and barrier [4]. In addition, oxidative stress aging is one of the key theories of skin aging related research [5]. Due to the formation of terminal glycosylation products (free radical peroxidation) on the collagen surface, the skin loses elasticity, resulting in the loss of elasticity of the skin's half bridging texture structure, and the flattening of the epidermal dermal connection, resulting in the skin becoming loose and inelastic [6]. Differences in skin inflammation at different ages lead to differences in skin defense systems [7]. Finally, inhibiting tyrosinase activity of melanocytes, promoting fibroblast proliferation, increasing the synthesis of collagen and hyaluronic acid, and inhibiting inflammation can delay skin aging [8].

In recent years, the theory of programmed aging has also attracted much attention. It mainly analyzes the aging phenomenon from the chromosome and genetic level [9]. Skin aging is mainly the result of increased expression of synthesis inhibition genes in chromosomal DNA and mitochondrial DNA of skin cells. Many genes related to cell activity are inhibited, and oxidative stress will damage DNA and affect its replication, transcription, and expression [10]. Therefore, gene regulatory factors may be the root of cell aging such as skin. SOX9 participates in high mobility family box transcription factors and plays a role in guiding tissue and cell morphogenesis, survival, and development. Relevant studies have shown that SOX9 is highly expressed in acne lesions [11]. In mice, the lack of SOX9 in early stem cells impedes hair follicle morphogenesis and epidermal wound repair [12]. More importantly, it is reported that tight junction proteins are also closely related to skin aging [13]. For example, the experiment of claudin expression disorder in epidermal cells confirmed the importance of claudin in epidermal differentiation and barrier function [14]. In addition, the transcription factor SOX9 can regulate the expression of claudin-8 to promote the growth of osteosarcoma cells [15]. However, there is no study on the effect of SOX9 regulating claudin 2 in keratinocytes on skin aging.

Since the skin is exposed to the surface, it is helpful to study the aging of the body at the molecular and cellular levels. In this study, the effects of transcription factor SOX9 on skin aging related factors, including keratinization, antioxidants, inflammatory mediators, and melanin deposition, were explored. Furthermore, the expression of SOX9 in normal epidermal keratinocytes and mice of different ages was determined. At 8 weeks and 24 months in vivo, SOX9 was strongly positively correlated with claudin 2. Overexpression of SOX9 could induce claudin 2 promoter activity in vitro. In addition, claudin 2 and SOX9 have similar effects on skin aging related factors. The results showed that claudin 2 was closely related to SOX9, and both claudin 2 and SOX9 were closely related to the process of skin aging.

This paper is organized as follows.  Section 2 discusses the related work, followed by the proposed methods in Section 3. In Section 4, the results and analysis are proposed. Finally, in Section 5, some concluding remarks are made.

## 2. Related Work

Skin aging is a developing, dynamic, slow, and complex physiological evolution process. The specific manifestations are skin relaxation, loss of elasticity, dry skin, and visible wrinkles. All these have seriously affected the external beauty of the skin and have become a topic of constant concern [16]. As the largest organ of the body, the skin becomes the most obvious manifestation of aging due to its bare surface [17]. Therefore, skin provides an excellent reference for the study of aging at the molecular and cellular levels.

Previous studies have shown that SOX9 is an important regulator of epidermal keratin-forming cells with recognized pro-proliferative and/or prosurvival functions that may be associated with several skin diseases characterized by abnormal differentiation and proliferation [18]. The aging of the skin surface is reflected at the cellular level as cellular senescence, which means that normal cells have only a certain life cycle and cannot proliferate indefinitely [19, 20]. The keratin-forming cells are the most dominant structural cells of the epidermis and are, from the inside out, the basal, spiny, granular, hyaline, and stratum corneum layers [21]. In the process of natural aging, the proliferation and differentiation of keratinocytes play an important role in regulating the formation of skin barrier and skin microenvironment [22]. Low expression of SOX9 is accompanied by a disturbing skin microenvironment. Together, SOX9 expression in keratinocytes may be associated with cellular senescence, which in turn is characterized by skin aging.

SOX9 acts as a transcription factor that binds to cis-acting elements of eukaryotic genes for specific interaction and regulation of gene transcription [23]. Overexpression of SOX9 activates the full-length promoter of claudin 2 in a dose-dependent manner. The frequency of base occurrences predicted from the JASPAR database requires focusing the core site of SOX9 regulation of claudin 2 transcriptions to -856 to -848 downstream of the claudin 2 promoters. SOX9 cis-response element deletion experiments on the claudin 2 promoter indicate that the core site of SOX9 regulation of claudin 2 transcription was at −856 to −848, consistent with the frequency of base occurrences predicted by JASPAR.

Claudin 2 is a member of the claudin family, the most important transmembrane protein among the many tight junction-related proteins. Tight junctions are a common form of intercellular junctions, which are found in epithelial, endothelial, and mesothelial cells, maintaining the polarity and barrier function of epithelial cells 14. For example, claudin-1, claudin-3, and claudin-7 protein and mRNA expression are significantly reduced in plaque psoriasis lesions. Lee et al. [24] reported a progressive decrease in claudin-1 expression from normal skin to photoaging keratosis. In the study, claudin 2 expression levels were lowest in the skin of newborn mice, peaking at around the 8th week and then decreasing with age. The expression of claudin 2 in different mouse skin tissues was consistent with the trend of SOX9. There was a significant difference in claudin 2 in skin tissues between 8-week-old mice and 24-month-old mice. Similarly, 24-month-old mice had elevated skin proinflammatory mediators, weakened antioxidant capacity, abnormal keratinocyte differentiation gene mRNA, and deposits of melanin. The low expression of SOX9 and the low expression of claudin 2 were consistent with the aging process of mouse skin. Therefore, claudin 2 may be involved in the aging process of the skin [25, 26].

Environmental factors also play a critical role in skin aging and can accelerate the normal physiological aging process of the skin. Ambient particulate matter (PM) can negatively affect human skin and exacerbate preexisting skin conditions [27]. PM2.5 induces keratinocytes to establish a model of cellular senescence and triggers overexpression of inflammation-related mediators TNF-*α*, IL-1*β*, IL-6, and COX-2 [28]. In addition, inflammatory reactions can occur from skin damage caused by high-intensity UV (ultraviolet) [29]. What is more, epidermal keratin-associated protein is the main epidermal structural protein that affects the function of the epidermal skin barrier [30]. KRT5/KRT14 in the basal layer of the epidermis is gradually replaced by KRT1/KRT10 as keratin-forming cells continue to differentiate terminally upwards, and KRT1/KRT10 begins to be expressed in the spiny layer, eventually replacing KRT5/KRT14 almost completely above the granular layer [31]. Mutations in keratin can affect the integrity of epidermal keratin-forming cells and thus cause epidermolysis bullosa [32]. Recombinant loricrin (Lor) is also important for cytoskeleton formation in the late stage of keratinization [33]. Furthermore, the body produces too much reactive oxygen species (ROS), which exceeds the body's clearance rate, and the oxidative and antioxidant systems become imbalanced [34]. Excess ROS participate in intracellular reactions, causing oxidative stress, a decrease in GSH-Px and SOD, and an increase in MDA [35]. Oxidative stress causes the loss of expression activity of genes that maintain essential cellular physiological functions through damage to DNA, which in turn leads to cellular senescence [36, 37]. Both EDN1 and PGE2 are closely related to the formation of melanin. Moreover, melanin is one of the remarkable features of aging [38]. Relevant studies have shown that PM2.5 induces the increase of inflammatory mediators, the decrease of antioxidant capacity, the abnormal mRNA of keratin differentiation genes, and melanin deposition in keratinocytes (NEK). After silencing claudin 2, overexpression of Sox9 lost its function. This indicates that the function of Sox9 in the aging process of keratinocytes may be closely related to claudin 2.

## 3. Proposed Methods

### 3.1. Animals and Grouping

C57BL/6 mice were housed individually (*n* = 6) per cage in the same environment for 12 hours alternating day and night, with free access to food and water and sterilized bedding changed three times a week, without adverse effects. Mice grow and age normally. Neonatal to 24-month-old mice were used to study skin aging, and all animals were injected intraperitoneally with 1% pentobarbital sodium (50 mg/kg) before cervical dislocation to obtain skin tissue for the next experiments. All experimental procedures were performed following the guidelines of experimental animals from Southwest Medical University. All animal experiments complied with the ARRIVE guidelines and in accordance with the U.K. Animals (Scientific Procedures).

### 3.2. Microarray Data Collection and Data Analysis

Skin tissues from 8-week-old and 24-month-old mice were collected for transcriptome sequencing. After RNA extraction, purification, and library construction, the skin tissue was assayed for insert size using an Agilent 2100 Bioanalyzer. The libraries were sequenced by Next-Generation Sequencing (NGS) technology, based on the Illumina sequencing platform, with Paired-end (PE) sequencing (the process was commissioned from Beijing Novozymes Technology Co.).

Transcriptome sequencing data were subjected to data quality control and sequence alignment to reference genes. Gene expression levels were quantified, and data were collated and filtered for differential gene analysis using edge R in R language software, using corrected *P* < 0.01 and log2 (fold change) >2 as thresholds for significant differential expression, to filter for differential genes between groups. The R language ggplots2 was used to map the volcanoes of differentially expressed genes, and the R language Pheatmap was used to obtain a heat map of the top 20 differential genes using a two-way cluster analysis of the concatenated sets of differential genes and samples from all comparison groups.

### 3.3. Cell Culture

Normal epidermal keratinocytes (NEK) and normal epidermal melanocytes (NEM) from mouse skin were purchased from YaJi Biological (Shanghai, China) [39]. Cell culture dishes were treated with poly-lysine (BI, Israel) and 10% FBS/DMEM with 100 U/mL penicillin and 100 g/mL streptomycin (BI, Israel) was used to culture NEK and NEM. The coculture of NEK and NEM is the same as that of the separate culture, with a ratio of 1 : 1. Keratinocytes were incubated with PM2.5 (50 ppm) for 72 h or keratinocytes in the upper chambers were pretreated with coculture medium containing PM2.5 (50 ppm) for 24 h and then perform target gene transfection and interfering sequence transfection for 24 h.

### 3.4. Transfection Assay

The si-RNA sequences involved in this experiment are as follows: si-claudin 2–1#: CACTGTGAGCTTGAGAGCTTCTCAA, si-claudin2–2#: GCACAGGCAGCAGAG TCCATTCTTA, si-claudin2–3#: GAGGCTGATGATGGGAGCATCTATT (Genepharma, China) [40]. The core sequence of SOX9 with claudin 2 was obtained by JASPAR (https://jaspar.genereg.net/) prediction. Different lengths of claudin 2 promoter plasmids were obtained by gradient deletion of SOX9 response elements. The plasmids in this experiment were all constructed by Shanghai Biotech. The vector for different lengths of claudin 2 promoter plasmids was pSI-Check2, carrying the ampicillin resistance gene. In addition, the vector for pc-DNA-SOX9 and pc-DNA-claudin 2 is pc-DNA3.1 with the kanamycin resistance gene.

These plasmids and interfering sequences were incubated for 20 min at room temperature using lipofectamine 2000 2000 (Invitrogen, Waltham, MA, USA) and serum-free medium [41]. Before transfection, the experimental cells were all replaced with fresh medium, followed by the addition of mixed liposome-coated plasmids and interfering sequences.

### 3.5. Reverse Transcriptase-Polymerase Chain Reaction (qRT-PCR)

Cells and skin tissue were collected and stored at −80°C. Total RNA was collected by the TRIzol RNA extraction kit (Invitrogen, USA) [42]. The integrity and purity of the RNA were determined by gel electrophoresis and NanoDrop 2000 spectrophotometry (Thermo, USA). Reverse transcription was performed using a reverse transcription kit (Invitrogen, USA) as described by the manufacturer. The resulting cDNA was quantified by qRT-PCR and evaluated using a Qubit fluorescence spectrometer (Invitrogen, USA) [43, 44].

### 3.6. Immunofluorescence Assay

Mouse skin tissue was collected and washed in saline and fixed overnight in 4% paraformaldehyde. Next, the tissue was dehydrated, paraffin-embedded, and made into sections. The slides were then blocked with 2% BSA for 30 min, and a primary antibody against SOX9 (1 : 300) was added and incubated overnight. After three piles of washing, the secondary antibody ALexaFluor-594 (Invitrogen, USA) was added for 2 hours. Finally, DAPI was used for nuclear staining of the cells. The slides were observed and photographed with a DM2000 fluorescence microscope (Leica, Germany) [45].

### 3.7. Immunohistochemistry Assay

Paraffin sections of mouse skin tissue were routinely dewaxed to water, thermally repaired with sodium citrate buffer antigen, inactivated at room temperature in 3% H_2_O_2_, and washed 3 times in PBS. SOX9 primary antibody was added at appropriate dilution (1 : 300) dropwise for 60 minutes at room temperature, and slices were washed 3 times with PBS. The appropriate amount of reaction enhancer dropwise was added for 20 min at room temperature, and slices were washed 3 times with PBS. An appropriate amount of horseradish enzyme-labeled goat anti-mouse IgG polymer (Shenggong BBILIFE, China) was used to incubate the sections for 20 min at room temperature and washed 3 times in PBS. DAB color development and light counterstaining with hematoxylin (Yeason, China) were dehydrated, transparent, mounted, and observed under the microscope. The brown particles in the cytoplasm were positive.

### 3.8. Western Blot Assay

Total proteins were extracted from cells or skin tissue, separated by SDS polyacrylamide gel electrophoresis, and electrostatically transferred to PVDF membranes. Membranes were closed with 5% skimmed milk TBS (50 mM Tris, pH 7.6, 0.9% NaCl, and 0.1% Tween-20) at room temperature and then incubated with primary antibodies for TNF-*α*, IL-1*β*, IL-6, and COX-2 (Abcam, UK) at 4°C overnight. The membrane was washed with TBS and then conjugated with HRP-labelled secondary antibody. After washing again, the protein bands were observed with Western ECL substrate (BIO-RAD, USA), and the results were determined using Image Lab software (BIO-RAD, USA) [46].

### 3.9. Flow Cytometry for ROS

1 × 106 cells of each group were washed twice in PBS. The cells were loaded with probes, prepared as 500 *μ*l of suspension cells containing 5 *μ*mol/L DCFH-DA (MCE, USA), reacted for 30 minutes at 37°C in the dark, and washed twice with PBS. The FITC channel was selected to analyze the changes of ROS in different groups.

### 3.10. Dual-Luciferase Reporter Assay

Cells transfected with target genes and interfering sequences were collected, lysed for 20 minutes using lysis solution, and the supernatant collected. 100 uL of supernatant was added into the 96-well full white enzymatic plate as reaction substrate. Next, 100 uL of firefly luciferase was added to each well via the autosampler (SpectraMax i3, USA), followed by the termination solution and 100 uL of Renilla luciferase (Promega, Madison, WI, USA) [47]. The ratio of firefly luciferase to Renilla luciferase was used as a reference for promoter activity.

### 3.11. Enzyme Linked Immunosorbent Assay (ELISA)

Mouse skin tissue or treated cells were collected and lysed with the appropriate amount of lysis solution. After this step, the supernatant was collected for ELISA testing [48]. MDA, GSH-Px, SOD, TNF-*α*, IL-1*β*, IL-6, COX-2, EDN1, and PGE2 were measured using the ELISA kit (Abcam, UK) according to the instructions [49]. Briefly, samples were added to a 96-well plate precoated with antibody (reaction substrate) and after several incubation steps, washing procedures, and final incubation with the chromogenic substrate, and the results were measured using an enzyme marker (Bio-Rad, USA).

### 3.12. Statistical Analysis

The experimental data were analyzed by SPSS21.0 software, and the measurement data were expressed as mean ± standard deviation ($\bar{x}$ ± *s*). Statistical comparisons were performed using one-way analysis of variance (ANOVA) and least-significant difference (LSD) post hoc for differences among multiple groups and an unpaired *t*-test for differences between two groups. *P* < 0.05 was considered to indicate a statistically significant difference.

## 4. Results and Analysis

### 4.1. Transcriptome Sequencing Analysis of Differential Gene Expression in Skin Tissues of Mice of Different Ages

Figure 1 showed the differential gene expression in skin tissues of 8-week-old and 24-month-old mice. Skin tissues from 8-week-old and 24-month-old mice were collected for transcriptome sequencing, and total RNA from mouse skin tissues was extracted for upsequencing and clustering analysis to obtain a volcano plot and heat map, as shown in Figure 1(a). Volcano plot results showed that 519 genes (red dots) were upregulated, and 1120 genes (blue dots) were downregulated in the skin tissue of 24-month-old mice compared with sequencing results of 8-week-old mice, but most genes (grey dots) did not show differences, as shown in Figure 1(b). The heat map results demonstrate the top 20 differential genes, with 11 genes upregulated and 9 genes downregulated in the skin tissue of 24-month-old mice compared with the 8-week-old mice sequencing results, with transcription factor SOX9 significantly downregulated, as shown in Figure 1(c).

### 4.2. Differential Expression of SOX9 in Skin Tissues of Mice of Different Ages

SOX9 was screened from the transcriptome sequencing results, and the expression of SOX9 was examined in the skin tissues of mice of different ages during growth and development. SOX9 mRNA levels in mouse skin tissue increased and then decreased from birth to 24 months.  Figure 2 showed the expression of SOX9 in skin tissues of mice from birth to 24 months. The results suggested that the involvement of SOX9 in the skin aging process may involve the involvement of keratinocytes cells. The expression level of SOX9 mRNA in newborn mice increased with growth and development, reaching a peak at about the 8th week, and then showed a downward trend, as shown in Figure 2(a). Immunofluorescence results showed low levels of SOX9 expression in the skin of newborn mice, with the highest levels at 8 weeks, and a significant decrease at 24 months of age. Immunofluorescence results showed low levels of SOX9 expression in the skin of newborn mice, with the highest levels at 8 weeks, and a significant decrease at 24 months of age, as shown in Figure 2(b). Immunohistochemical showed that SOX9 at different ages coincided with mRNA and immunofluorescence, and SOX9 was mainly concentrated in keratinocytes cells in the skin, as shown in Figure 2(c).

### 4.3. Effects of SOX9 on PM2.5-Induced Keratinocyte Cells

Overexpression of SOX9 and a model of premature skin aging induced by particulate matter (PM2.5) were used to further investigate the effects of SOX9 and keratinocyte cells on the skin aging process.  Figure 3 demonstrated the regulation of oxidative stress, differentiation, inflammation, and melanin deposition in NEK by SOX9. The results revealed that SOX9 on the skin aging process may be related to keratinocyte formation, inflammation, antioxidation, and melanin deposition. SOX9 mRNA was able to be significantly upregulated by pcDNA-SOX9, as shown in Figure 3(a). Compared with the blank group, Krt1 and Krt10 were reduced in the PM2.5 induction group, and Krt14 and Lor were increased under the PM2.5 induction group. Compared with the PM2.5-induced group, pcDNA-NC did not affect Krt1, Krt10, Krt14, and Lor, whereas pcDNA-SOX9 upregulated Krt1 and Krt10 and downregulated Krt14 and Lor, as shown in Figure 3(b). In addition, the inflammatory mediators TNF-*α*, IL-1*β*, IL-6, and COX-2 were significantly increased in NEK under the effect of PM2.5 compared with the blank group. Compared with the PM2.5-induced group, pcDNA-NC had no significant effect on these inflammatory mediators, while pcDNA-SOX9 suppressed the levels of these inflammatory mediators, as shown in Figure 3(c). ROS was correlated with cellular antioxidant capacity and was significantly increased in NEK cells under PM2.5 induction compared with the blank group, while pcDNA-SOX9 could inhibit ROS, and pcDNA-NC had no effect, as shown in Figure 3(d). Finally, melanin deposition was closely associated with skin aging, and NEK and NM cocultures were used to verify the effect of SOX9 in melanin formation. Compared with the blank group, PM2.5 induced a significant increase in EDN1 and PGE2 in NEK cells, while pcDNA-SOX9 could inhibit the induction of PM2.5, while pcDNA-NC had no effect, as shown in Figure 3(e).

### 4.4. Effect of SOX9 on Claudin 2 Promoter Activity

Bioinformatics predicted that claudin 2 could be regulated by SOX9. By using JASPAR software, a construct containing the upstream promoter region of claudin 2 (−2.0 kb) is performed to predict the cis-response element of SOX9 and the binding site of the claudin 2 promoter.  Figure 4 showed that SOX9 regulates claudin 2 promoter activity in HEK-293 cells. SOX9 response element at the promoter can be illustrated in Figure 4(a). The effect of SOX9 on claudin 2 promoter activity was further verified using a luciferase assay. Overexpression of SOX9 had a dosage effect on activation of the claudin 2 promoter, as shown in Figure 4(b). In contrast, the disordered pcDNA-NC did not affect claudin 2 promoter activity, and the vacant plasmids (PSI-NC) did not respond to overexpression of SOX9, as shown in Figure 4(c). Finally, the results of promoter truncation experiments indicate that the presence of a SOX9 response element at −856 upstream of the claudin 2 promoter appears to have little effect on claudin 2 transcription, while −856 to −848 (GTTGTTACT) may be an important binding site. Groups represented by different letters have significant differences at *P* < 0.05, while the same letters indicate no significant differences. The results confirm that SOX9 can activate the claudin 2 promoter, and the interaction should exist between SOX9 and claudin 2.

### 4.5. Effects of Claudin 2 on PM2.5-Induced Keratin-Forming Cells

SOX9 could regulate claudin 2 promoter activity, and the effect of claudin 2 on the senescence process was verified using overexpressed and knocked out claudin 2.  Figure 5 demonstrated the regulation of oxidative stress, differentiation, inflammation, and melanin deposition in NEK by claudin 2. The levels of claudin 2 mRNA during mouse growth and development were relatively consistent with the trend of SOX9, both increasing and then decreasing, reaching a peak at about the 8th week, as shown in Figure 5(a). In NEK cells, claudin 2 was induced by pcDNA-claudin 2, as shown in Figure 5(b). And it also was inhibited by si-claudin 2, with si-claudin 2–2# being the most efficient inhibitor, as shown in Figure 5(c). Therefore, si-claudin 2–2# was the next subject of study. PcDNA-SOX9, pcDNA-claudin 2, and si-claudin 2–2# were transfected separately or cotransfected to detect whether SOX9 affects keratinocyte state by regulating claudin 2. Compared with the blank group, Krt1 and Krt10 were inhibited by PM2.5, and Krt14 and Lor increased. Compared with the PM2.5 group, pcDNA-SOX9 and pcDNA-claudin 2 could restore the downregulation of Krt1 and Krt10 and suppress the expression of Krt14 and Lor. In contrast, pcDNA-SOX9 and si-claudin 2–2# did not affect the adverse induction of PM2.5, as shown in Figure 5(d). Flow cytometry results showed that pcDNA-SOX9 and pcDNA-claudin could inhibit PM2.5-induced ROS levels, while pcDNA-SOX9 in concert with si-claudin 2–2# had no effect, as shown in Figure 5(e). Similarly, pcDNA-SOX9 and pcDNA-claudin 2 could inhibit PM2.5-induced inflammatory mediators (TNF-*α*, IL-1*β*, IL-6, and COX-2), whereas pcDNA-SOX9 in concert with si-claudin 2–2# was ineffective, as shown in Figure 5(f). Finally, pcDNA-SOX9 and pcDNA-claudin 2 could inhibit PM2.5-induced EDN1 and PGE2, whereas pcDNA-SOX9 in concert with si-claudin 2–2# had no effect (Figure 5(f)). These results suggested that pcDNA-SOX9 and pcDNA-claudin 2 had similar or synergistic effects in NEK. Besides, the effect of pcDNA-SOX9 was counteracted by si-claudin 2–2#, indicating that SOX9 was closely related to claudin 2 in NEK.

### 4.6. Differential Factors in Skin Tissue of Mice of Different Ages

Figure 6 showed the differences in oxidative stress, keratinocyte differentiation, inflammation, and melanin deposition in the skin tissues of 8-week-old and 24-month-old mice. There was a strong positive correlation between SOX9 and claudin 2 levels in the skin of both 8-week-old and 24-month-old mice, as shown in Figures 6(a) and 6(b). The skin tissue of 24-month-old mice showed increased MDA, decreased GSH-Px and SOD, and reduced antioxidant capacity, as shown in Figure 6(c). Furthermore, Krt1 and Krt10 were reduced, and Krt14 and Lor were increased in 24-month-old mice compared with 8-week-old mice, as illustrated in Figure 6(d). Proinflammatory mediators (TNF-*α*, IL-1*β*, IL-6, and COX-2) were significantly higher in 24-month-old mice compared with 8-week-old mice, with inflammatory infiltration of skin tissue, as shown in Figure 6(e). EDN1 and PGE2 were more abundant in the skin tissue of 24-month-old mice with melanin deposition compared with 8-week-old mice, as shown in Figure 6(f). The results suggest that the differences in various indicators in the skin of 8-week-old versus 24-month-old mice may be related to differences of SOX9 and claudin 2 Primer designs were obtained from NCBI (https://www.ncbi.nlm.nih.gov/) (Table 1).

## 5. Conclusion

In this study, the skin of 8-week-old and 24-month-old mice is sequenced to obtain a differentially expressed gene SOX9. Our results can provide effective evidence that Sox9 and claudin 2 are involved in the process of skin aging. SOX9 could regulate claudin 2 transcription in vitro, and in vivo SOX9 has a strong positive correlation with claudin 2 levels. In addition, the ability of SOX9 to retard PM2.5-induced premature aging models appears to involve claudin 2. In the future, we will further study the possible synergy between pcdna-sox9 and pcDNA-claudin 2.

## Figures and Tables

**Figure 1:** Differential gene expression in skin tissues of 8-week-old and 24-month-old mice: (a) library building and sequencing process; (b) volcano plot of differentially expressed genes; (c) heat map of the top 20 differential genes.

**Figure 2:** The expression of SOX9 in skin tissues of mice from birth to 24 months: (a) the mRNA expression of SOX9; (b) immunofluorescence for SOX9; (c) immunohistochemistry for SOX9.

**Figure 3:** Regulation of oxidative stress, differentiation, inflammation, and melanin deposition in NEK by SOX9: (a) expression of SOX9 in NEK; (b) Krt1, Krt10, Krt14, and Lor in NEK; (c) TNF-*α*, IL-1*β*, IL-6, and COX-2 in NEK; (d) Regulation of ROS by SOX9 in NEK; (e) EDN1 and PGE2 in NEK and NM. Groups represented by different letters have significant differences at *P* < 0.05, while the same letters indicate no significant differences.

**Figure 4:** SOX9 regulates claudin 2 promoter activity in HEK-293 cells: (a) SOX9 response element at the promoter; (b) dose relationship of SOX9 on claudin promoter activity; (c) schematic representation of the claudin 2 5′ upstream promoter region, and SOX9 binds to the claudin2 promoter binding site (pcDNA-SOX9, 100 ng).

**Figure 5:** Regulation of oxidative stress, differentiation, inflammation, and melanin deposition in NEK by claudin 2: (a) expression of claudin 2 in the skin of mice of different ages; (b) activation of claudin 2 in NEK; (c) inhibition of claudin 2 in NEK; (d) Krt1, Krt10, Krt14, and Lor in NEK; (e) regulation of ROS by claudin 2 in NEK; (f) TNF-*α*, IL-1*β*, IL-6, and COX-2 in NEK; (g) EDN1 and PGE2 in NEK and NM.

**Figure 6:** Differences in oxidative stress, keratinocyte differentiation, inflammation, and melanin deposition in the skin tissues of 8-week-old and 24-month-old mice: (a) scatter plot of correlation analysis between SOX9 and claudin 2 at 8 weeks, *Y* = 1.652*∗X* − 4.520, *R*^2^ = 0.7453; (b) scatter plot of correlation analysis between SOX9 and claudin 2 at 24 months, *Y* = 0.7862*∗X* + 0.4914, *R*^2^ = 0.7372; (c) oxidative stress-related factors MDA, GSH-Px, and SOD; (d) Skin keratin formation-related genes Krt1, Krt10, Krt14, and Lor; (e) inflammatory mediators TNF-*α*, IL-1*β*, IL-6, and COX-2; (f) melanogenesis-related factors EDN1 and PGE2.

**Table 1:** Primer sequences.

Gene	Primer sequences
*β*-actin	F: GAAGATCAAGATCATTGCTCC
	R: TACTCCTGCTTGCTGATCCA
Krt1	F: CATGGAGATTGCCACATACAAG
	R: GCTACTGCTTCCGCTCAT
Krt10	F: GATGCTGAAGAGTGGTTCAATC
	R: TCAGACTTATGGCTGGACATTT
Krt14	F: CTACCTGAAGAAGAACCACGAG
	R: CATCTTCTCGTACTGATCCCG
Lor	F: CTGTGGGTTGTGGAAAGACCTCTG
	R: CAGCTAGAGCCTCCTCCAGATGAG
SOX9	F: GAGTTTGACCAATACTTGCCAC
	R: ACTGCCAGTGTAGGTGAC
Claudin 2	F: GGTTCCTGACAGCATGAAATTT
	R: GCCATCATAGTAGTTGGTACGA

## Data Availability

The datasets used or analyzed during the current study are available from the corresponding author upon reasonable request.
